The article "Rabbiteye blueberry prevents osteoporosis in ovariectomized rats" was published in 2014. Journal: J Orthop Surg Res.

# Rabbiteye blueberry prevents osteoporosis in ovariectomized rats

**DOI:** 10.1186/s13018-014-0056-9

**Published:** 2014-08-08

**Authors:** Tao Li, Shou-Mian Wu, Zhi-Yuan Xu, Sheng Ou-Yang

**Affiliations:** 1 Department of Orthopedics, The Third Affiliated Hospital of Southern Medical University (Academy of Orthopedics), Guangzhou 510630, Guangdong Province, China; 2 Department of Emergency, The Third Affiliated Hospital of Southern Medical University, Guangzhou 510630, China

**Keywords:** Rabbiteye blueberry, Osteoporosis, Alkaline phosphatase activity, Focal adhesion kinase, Bone histomorphometry

## Abstract

**Objective:**

It has been forecasted that the rabbiteye blueberry could inhibit osteoporosis. However, the inhibition and prevention of osteoporosis via rabbiteye blueberry are still elusive. This study was aim to evaluate the anti-osteoporosis effects of rabbiteye blueberry in ovariectomized rats.

**Methods:**

Thirty rats were randomly divided into three groups of ten rats each as follows: sham-operated group (SG), ovariectomized model control group (OMG), and ovariectomized rabbiteye blueberry treatment group (OBG). The blood mineral levels, the alkaline phosphatase (ALP) activity, and osteoprotegerin (OPG) level were determined. The expression analyses of type I collagen, integrin-β1, and focal adhesion kinase (FAK) were performed. Besides, the bone mineral density (BMD) and bone histomorphometry (BH) were measured.

**Results:**

The ALP activity in SG and OBG was significantly lower than that in OMG. For the OPG level, the significant increase of OPG level in OBG was indicated compared with the other groups. The mRNA expression levels of type I collagen, integrin-β1, and FAK in OMG were significantly lower than those in other groups. The BMD in OMG were all significantly lower than those in SG and OBG. For BH, blueberry significantly improved the trabecular bone volume fraction, trabecular thickness, mean trabecular bone number, and bone formation rate, and decreased the trabecular separation, the percent of bone resorption perimeter, and mean osteoclast number in OBG compared with OMG.

**Conclusions:**

The rabbiteye blueberries had an effective inhibition in bone resorption, bone loss, and reduction of bone strength of ovariectomized rats and could improve the BMD, osteogenic activity, and trabecular bone structure.

## Introduction

Osteoporosis is a systemic skeletal disease characterized by low bone mass and microarchitectural deterioration of bone tissue, with a consequent increase in bone fragility and susceptibility to fracture [1]. In the USA, there are 10 million Americans with osteoporosis (8 million women and 2 million men) and another 34 million individuals with osteopenia, which resulted in a significant proportion of the population to be deemed ‘at risk’ [2].

The article "Rabbiteye blueberry prevents osteoporosis in ovariectomized rats" was published in 2014. Journal: J Orthop Surg Res.

The major current anti-osteoporotic therapy is pharmacologic treatment including bisphosphonates, estrogens, selective estrogen receptor modulators, and parathyroid hormone [3]. In the past 5 years, additional drugs were likely to have been approved, such as the anti-RANK ligand monoclonal antibody [4] and cathepsin K inhibitors [5]. Most of the pharmacologic therapy strategies have been adopted that aim to inhibit excessive bone resorption and increase bone formation. There were also managements focused on non-pharmacologic treatments, such as a balanced diet and adequate calcium and vitamin D intake [6]. Folic acid [7], vitamin B_12_[8], carotenoid [9], and lycopene [10] have been reported effective in improving bone loss and relieving the symptoms of osteoporosis in postmenopausal women [11].

Rabbiteye blueberry (*Vaccinium ashei* Reade) is a highly heterozygous, cross-pollinating fruit species, and belongs to the genus *Vaccinium* (*Vaccinium* spp.) and Ericaceae family. Recent reports showed that feeding a high-quality diet supplemented with blueberries to pre-pubertal rats or the rats at postnatal day 20 to 34 prevented ovariectomy-induced bone loss in adult life [12]. The molecular mechanisms underlying these effects may involve the increase of myosin production and reduction of mesenchymal stromal cell senescence. However, the effect of blueberry diet on inhibiting ovariectomy-induced osteoporosis and its mechanisms still need research.

In order to provide more evidence and gain a better understanding on the association between the active ingredients of rabbiteye blueberries and the inhibition of ovariectomy-induced osteoporosis, *in vivo* experiments on ovariectomized rat models have been conducted in this study. The blood mineral levels, the activity of alkaline phosphatase (ALP), and osteoprotegerin (OPG) level were determined to evaluate the effect of rabbiteye blueberry to osteoporosis. The expression analysis of type I collagen, integrin-β1, and focal adhesion kinase (FAK) was performed to explore the influence of rabbiteye blueberries on the osteoporosis-related integrin pathway. Further measurements of bone mineral density (BMD) and bone histomorphometry (BH) were performed to observe bone microstructure and dynamic changes of bone metabolism in osteoporosis.

## Materials and methods

### Experimental animals

Our experimental research on animals followed internationally recognized guidelines. The Animal Ethics Committee of Shanghai Jiao Tong University School of Medicine approved the study (reference number 2010–0018).

The article "Rabbiteye blueberry prevents osteoporosis in ovariectomized rats" was published in 2014. Journal: J Orthop Surg Res.

A total of 30 normal 8-week-old female Sprague–Dawley rats (160 ± 15 g) were provided by the Laboratory of Animal Science Department of Shanghai Jiao Tong University School of Medicine. The 30 rats were housed in ten cages with temperature of 21°C ± 1°C, relative humidity of 60%, ambient noise <50 dB, and regular 12-h light cycle. All rats were feed with conventional food and free access to water.

### Operative techniques

The 30 rats were randomly divided into three groups of ten rats each as follows: sham-operated group (SG), ovariectomized model control group (OMG), and ovariectomized blueberry treatment group (OBG). All rats were anesthetized before operation by intraperitoneal injection with 1% (volume fraction) pentobarbital sodium at a dose of 40 mg/kg. The operation begun through a 1-cm longitudinal incision at the back, 1 cm from the spine and 2 cm above the posterior iliac crest. Bilateral oophorectomy was performed on the rats of OMG and OBG, while same weights of greater omentums were removed instead of ovary for the rats of SG. Finally, the wound was closed in layers after stump ligation.

### Rabbiteye blueberry administration

After the operation, penicillin was intramuscularly injected to all the rats for three consecutive days. One week later, the rats in the OBG were administered with freeze-dried blueberry powder water solution (10%, *w*/*w*) for 12 consecutive weeks by gavage, while the rats in the SG and OMG were administered with equal volume of double distilled water by gavage. The freeze-dried blueberry powder (stored at −20°C) was provided by the Institute of Botany, Chinese Academy of Sciences, Beijing, China.

### Determination of the levels of serum minerals, ALP, and OPG

After the 12-week administration, the rats were anesthetized by intraperitoneal injection of 20% (*w*/*v*) urethane solution at a dose of 1 mg/kg. The blood samples were collected from the abdominal aorta and then the serum was obtained by centrifugation at a low temperature of 4°C. The levels of the serum minerals were determined by using an automatic biochemical analyzer. The ALP activity was determined using an Alkaline Phosphatase Opt Kit (Roche Molecular Biochemical, Indianapolis, IN, USA). The OPG level in serum was measured by ELISA using the Biomedical rat OPG ELISA kit (Biomedical, Wien, Austria). All measurements were performed according to the manufacturer’s instructions.

### Total RNA extraction and reverse transcription of RNA

After being fasted for 24 h, all the rats were sacrificed. Then, the third lumbar vertebra without surrounding soft tissues was quickly collected at once. After homogenized treatment, the total RNA was extracted by using Trizol Reagent (Shanghai Jianglai Biotechnology Co., Ltd., Shanghai, China) according to the manufacturer’s recommendations. The quantity and quality of RNA were determined by UV absorbance at 260-, 280-, and 320-nm wavelengths using NanoDrop ND-1000 (Thermo Fisher Scientific Inc., Waltham, MA, USA). Complementary DNA (cDNA) was synthesized from RNA using Reverse-transcription kit (Life Technologies Company, Beijing, China) with Superscript II Reverse Transcriptase (Life Technologies Inc., CA, USA) according to the manufacturer’s recommendations.

The article "Rabbiteye blueberry prevents osteoporosis in ovariectomized rats" was published in 2014. Journal: J Orthop Surg Res.

### Detection of expression of type I collagen, integrin-β1, and focal adhesion kinase

The real-time quantitative polymerase chain reaction (PCR) was carried out by CFX96 Real-Time PCR instrument (Bio-Rad, Hercules, CA, USA). SYBR Green I was provided by Shanghai Life Technology Company (Shanghai, China). Primers of *collagen-1* (encoding type I collagen), *integrin-β1* (encoding integrin-β1), *FAK* (encoding focal adhesion kinase), and *β-actin* were shown in Table 1. The real-time quantitative PCR was carried out under the following conditions: preheating at 95°C for 5 min, followed by 45 cycles of denaturation at 95°C for 1 min, annealing at 54°C for 1 min, and extension at 74°C for 2 min. The PCR amplification was ended by a final extension cycle at 72°C for 10 min. After obtaining the amplification curve and the CT values, the dissolve curve was analyzed using the following setting: 95°C for 15 s, 60°C for 1 min, and 95°C for 15 s. The relative expression of each biomarker was represented as the radio of the copy number of each sample and *β-actin*.

**Table 1:** **Primers of** ***collagen-1*,** ***integrin-β1*,** ***FAK*, and** ***β-actin***

**Gene name**	**Forward primer**	**Reverse primer**
*Collagen-1*	ATCAAGGTCACTGCAACAT	CAGGATCAAACCTTCGCTT
*Integrin-β1*	CCCTTTCCTCAGAAGTCATTTTG	TTCGCTTTGGCATTCACATTCAC
*FAK*	CGGGATCCGCATCAGCATA	CCCAAGCTTTTAGTGCCTG
*β-actin*	TCT TCC AGC CTT CCT TCC TG	TAG AGC CAC CAA TCC ACA CA

*Collagen-1* encodes type I collagen, *integrin-β1* encodes integrin-β1, and *FAK* encodes focal adhesion kinase.

### Detection of BMD

The left femur BMD was measured by using EXA-3000 dual-energy X-ray BMD measure instrument (MEDILINK, Mauguio, France). Based on actual length measured by the measuring instrument, the left femur BMD was divided into three parts: the proximal BMD (pBMD) in the upper portion including one fourth of the femur, the middle (mBMD) in middle portion including one half of the femur, and the distance (dBMD) in the lower end portion including one fourth of the femur.

### Detection of histomorphometry

The complete right femur and tibia were used to prepare bone specimens for analyzing BH. The bone specimens were stained by von Kossa and Giemsa before they were observed and imaged by fluorescent/optical microscope (Leica DM4000B, Stuttgart, Germany). Randomly selected images in the inner, middle, and outer of the specimen were saved.

The article "Rabbiteye blueberry prevents osteoporosis in ovariectomized rats" was published in 2014. Journal: J Orthop Surg Res.

Static and dynamic histomorphometric measurements of the secondary cancellous bone located within 4.0 mm distal to the growth plate-metaphyseal were performed. The specimens stained with von Kossa were used for histology observation, while the specimens stained with Giemsa were used to observe osteoid. The data of BH were analyzed by using a color image analysis software of Leica.

### Statistical analysis

The SPSS 12.0 software (http://www-01.ibm.com/software/analytics/spss/) was used for the statistical analysis. The results were all expressed as mean ± SEM. The analysis of variance and multiple comparison tests were performed with *p* value less than 0.05, which was considered as significant.

## Results

### Serum mineral levels

The serum minerals were monitored for changes that may affect bone mineralization. The levels of serum minerals (Ca, P, and Mg) in each group were shown in percentages (Table 2). The results indicated that there was no significant difference in the levels of serum minerals (Ca, P, and Mg) among the three groups with *p* value of more than 0.05.

**Table 2:** The levels of serum minerals (Ca, P, and Mg) in each group

**Name**	**OMG**	**SG**	**OBG**
Ca (mmol/L)	2.20 ± 0.16	2.34 ± 0.08	2.22 ± 0.21
P (mmol/L)	1.62 ± 0.24	1.71 ± 0.17	1.82 ± 0.14
Mg (mmol/L)	0.63 ± 0.11	0.52 ± 0.08	0.53 ± 0.12

*OMG* ovariectomized model control group, *SG* sham-operated group, *OBG* ovariectomized rabbiteye blueberry treatment group.

### OPG level and ALP activity

The ALP activity in SG and OBG was significantly lower than that in OMG (SG vs. OMG: *p* = 0.035; OBG vs. OMG: *p* = 0.041), and there was no significant difference between SG and OBG. For the OPG level in the serum, the significant increase of OPG level in OBG was indicated when compared with the other groups (OBG vs. SG: *p* = 0.029). The OPG level in SG was significantly lower than that in OMG (Figure 1).

**Figure 1:** **The alkaline phosphatase (ALP) activity and osteoprotegerin (OPG) level in each group (*n*** **= 10).** The activity (right image) and level (left image) were compared with those in the ovariectomized model control group (*p < 0.05, **p < 0.01) and compared with those in the sham-operated group (#*p* < 0.05). Model: ovariectomized model control group (OMG); sham: sham-operated group (SG); blueberry: ovariectomized blueberry treatment group (OBG).

### The mRNA expression levels of type I collagen, integrin-β1, and FAK

Compared with the OMG, the mRNA expression levels of type I collagen, integrin-β1, and FAK were significantly higher in the OBG and SG (type I collagen: SG vs. OMG, *p* = 0.005; OBG vs. OMG, *p* = 0.001; integrin-β1: SG vs. OMG, *p* = 0.008; OBG vs. OMG, *p* = 0.001; FAK: SG vs. OMG, *p* = 0.008; OBG vs. OMG, *p* = 0.001). Moreover, their mRNA expression levels in OBG were significantly increased compared with those in SG (type I collagen: OBG vs. SG, *p* = 0.001; integrin-β1: OBG vs. SG, *p* = 0.001; FAK: OBG vs. SG, *p* = 0.001) (Figure 2).

The article "Rabbiteye blueberry prevents osteoporosis in ovariectomized rats" was published in 2014. Journal: J Orthop Surg Res.

**Figure 2:** **mRNA expression levels of type I collagen, integrin-β1, and FAK in each group (*n*** **= 10).** The levels were compared with those in the ovariectomized model control group (*p < 0.01) and compared with those in the sham-operated group (#*p* < 0.01). Model: ovariectomized model control group (OMG); sham: sham-operated group (SG); blueberry: ovariectomized blueberry treatment group (OBG).

### Comparison of BMD

The total BMD, pBMD, mBMD, and dBMD in OMG were all significantly lower than those in SG (total BMD: *p* = 0.012; pBMD: *p* = 0.025; mBMD: *p* = 0.016; dBMD: *p* = 0.021). Compared with the OMG, the total BMD, pBMD, mBMD, and dBMD were all significantly increased in OBG (total BMD: *p* = 0.028; pBMD: *p* = 0.036; mBMD: *p* = 0.045; dBMD: *p* = 0.042) (Figure 3).

**Figure 3:** **Bone mineral density of rats in each group (*n*** **= 10).** The BMD was compared with that in the ovariectomized model group (*p < 0.05). Model: ovariectomized model control group (OMG); sham: sham-operated group (SG); blueberry: ovariectomized blueberry treatment group (OBG).

### Bone histomorphology

The statistical analysis for the results of histomorphometric measurements indicated that the static and dynamic parameters of BH in SG and OBG presented significant differences compared with the OMG. The trabecular bone volume fraction (trabecular bone volume (BV)/total tissue volume (TV)), trabecular thickness (Tb. Th), and mean trabecular bone number (Tb. N) in OBG and SG were significant higher than those in OMG (*p* < 0.01). The trabecular separation (Tb. Sp), the percent of bone resorption perimeter (ES/BS), and the mean osteoclast number (Oc. N) in OBG and SG were significantly lower than those in OMG (*p* < 0.05). The osteoid perimeter (O. Pm) in SG was significantly lower than that in OMG (*p* < 0.05), while there was no significant difference in the osteoid perimeter between OBG and OMG. The fluorescent tag circumference ratio (L. Pm) was significantly lower in SG than in OMG (*p* < 0.01) but significantly higher in OBG than in OMG (*p* < 0.05). The bone formation rate (BFR/BV) in OBG and SG was higher than that in OMG (*p* < 0.01) (Table 3).

The article "Rabbiteye blueberry prevents osteoporosis in ovariectomized rats" was published in 2014. Journal: J Orthop Surg Res.

**Table 3:** Results of bone histomorphometry in each group

	**OMG**	**SG**	***p*** **value**	**OBG**	***p*** **value**
BV/TV (%)	16.38 ± 5.69	29.47 ± 6.52*	0.001	22.39 ± 5.26*	0.005
Tb. Th (μm)	48.96 ± 8.64	85.36 ± 9.35*	0.001	72.96 ± 7.37*	0.002
Tb. N (L/mm)	1.69 ± 0.16	2.05 ± 0.16*	0.005	1.89 ± 0.11*	0.008
Tb. Sp (μm)	763.85 ± 138.24	369.42 ± 102.34*	0.001	587.56 ± 185.21*	0.008
ES/BS (%)	18.27 ± 4.82	9.50 ± 4.42*	0.007	14.27 ± 4.23**	0.044
Oc. N (L/mm^2^)	0.26 ± 0.08	0.10 ± 0.06*	0.001	0.20 ± 0.05**	0.039
O. Pm (%)	30.35 ± 6.32	18.84 ± 6.47**	0.030	31.13 ± 5.08	-
L. Pm (%)	15.03 ± 1.26	8.63 ± 1.09*	0.001	16.98 ± 3.25**	0.041
BFR/BV (%/year)	36.85 ± 6.23	58.27 ± 7.03*	0.002	61.23 ± 13.91*	0.001

*p < 0.01 and **p < 0.05 compared with the OMG. *OMG* ovariectomized model control group, *SG* sham-operated group, *OBG* ovariectomized rabbiteye blueberry treatment group, *BV/TV* trabecular bone volume fraction (trabecular bone volume (BV)/total tissue volume (TV)), *Tb. Th* trabecular thickness, *Tb. N* mean trabecular bone number, *Tb. Sp* trabecular separation, *ES/BS* the percent of bone resorption perimeter, *Oc. N* mean osteoclast number, *O. Pm* osteoid perimeter, *L. Pm* fluorescent tag circumference ratio, *BFR/BV* bone formation rate.

## Discussion

Osteoporosis is a systemic skeletal disease that is often accompanied with a decrease of bone mass and microarchitectural deterioration of bone tissue, which can lead to an enhanced bone fragility and consequent increase in fracture risk [13]. The risk is greater in postmenopausal women due to deficiency of estrogen [14], which was considered the seminal mechanism of osteoporosis in both women and men [15]. Thus, a further understanding on osteoporosis pathogenesis, combined with the development of treatments with proven efficacy, will increase demand for the more effective management of patients with osteoporosis [16]. The lyophilized rabbiteye blueberries have been reported to have antioxidant activity [17] and can affect lipid metabolism [18]. In addition, it was reported that GTP supplementation plus alphacalcidol administration increased bone mass via a decrease of oxidative stress [19]. Therefore, its antioxidant activity may be one of the mechanisms for preventing osteoporosis. However, there are few studies focusing on the preventive effects of rabbiteye blueberries on postmenopausal osteoporosis which is the most common cause of age-related bone loss.

Ovariectomy-induced bone loss and postmenopausal bone loss in the rat share many similar characteristics [20]. Thus, the ovariectomy-induced osteoporosis in rat was used as a model for postmenopausal osteoporosis in humans in this study. Bone mineral mainly includes Ca, P, and Mg, and bone metabolism can be indirectly studied through their levels in the serum. In this study, their levels presented no significant difference among the three groups. The reason may be that the loss of bone mineral presents as a slow process due to a more active bone resorption than bone formation in the ovariectomized rats.

The article "Rabbiteye blueberry prevents osteoporosis in ovariectomized rats" was published in 2014. Journal: J Orthop Surg Res.

The ALP activity in the OMG presented a sharp rise compared with those in the other groups and no significant difference between OBG and SG, suggesting that the rabbiteye blueberry diet played a bone-protective role in the ovariectomized rat model. Moreover, the OPG level in OBG was significantly increased compared with those in the OMG and SG. It is well known that the balance between bone formation and bone resorption is essential for bone mass and bone microstructure [21]. ALP is assessed as a marker of bone formation [22], while OPG is identified as an inhibitor of osteoclastogenesis, osteoclast differentiation, and activation both *in vitro* and *in vivo*[23]. Significantly lower ALP activity and higher OPG level in OBG than in OMG were detected, revealing that rabbiteye blueberry can prevent osteoblast development by increasing the OPG level and can prevent osteoporosis by inhibiting the ALP activity.

Integrins are heterodimeric transmembrane proteins consisting of α and β subunits that functionally serve as both adhesive and signaling receptors [24]. Integrin-β1 is a major receptor of matrix glycoproteins in type I collagen-induced osteoblastic differentiation of bone marrow cells [25]. Type I collagen interacts with integrin-β1 receptor on the cell membrane, mediates extracellular signals into cells, and activates the FAK signal pathway. FAK is the immediate transducer in integrin-β1-dependent adhesion of osteoblasts to bone matrices [26]. In this study, we observed that the mRNAs of type I collagen, integrin-β1, and FAK in OMG expressed less than those in SG and OBG, and they expressed more in OBG than in SG. Ovariectomy could induce estrogen deficiency and increase bone resorption which led to accelerated collagen degradation and reduced collagen synthesis, especially type I collagen [27],[28]; then, the expression of integrin-β1 and FAK may be affected. The reason may be that the mRNA expression levels of type I collagen, integrin-β1, and FAK in the model rats were decreased in OMG. Meanwhile, the mRNA expression levels of type I collagen, integrin-β1, and FAK in OBG were significantly higher than those in the other groups, indicating that rabbiteye blueberry played a positive role in preventing osteoporosis. The integrin-β1/FAK signaling pathway may be repaired by active ingredients in blueberry to induce the increase of osteogenic activity.

The article "Rabbiteye blueberry prevents osteoporosis in ovariectomized rats" was published in 2014. Journal: J Orthop Surg Res.

Bone strength is determined by bone mass and bone quality. Bone mass is estimated in clinical practice by measuring the BMD. Menopause is the largest contributor to decreasing bone mineral density due to the significant decrease of estrogen [29]. The total BMD, pBMD, mBMD, and dBMD in OMG were all significantly lower than those in SG, and blueberry increased the BMD in OBG compared with OMG. This indicated that blueberry could effectively improve BMD of ovariectomized rats. Compared to BMD, BH can reflect the bone quality including bone microstructure and dynamic changes of bone metabolism. Trabecular bone belongs to cancellous bone, which is more sensitive to osteopenia than the cortical bone [30]. The trabecular architecture becomes more rod-like and anisotropic in osteoporotic and aging trabecular bone [31],[32], even completely disappears in postmenopausal women and ovariectomized rats [33]. In this study, rabbiteye blueberries significantly improved the trabecular bone volume fraction, trabecular thickness, and mean trabecular bone number, and decrease the trabecular separation in OBG compared with OMG. Thus, the active ingredients in blueberry could prevent the loss of trabecular bone in osteoporosis.

It was reported that the decrease of estrogen enhanced the osteoclast development and increased the number of osteoclasts in the trabecular bone [34]. According to the results of this study, the percent of bone resorption perimeter and mean osteoclast number in OBG and SG were significantly lower than those in OMG, and the bone formation rate in OBG and SG were higher than that in OMG, indicating that the blueberry effectively inhibited the development of osteoclast and bone resorption and promoted bone formation. However, the osteoid perimeter and the fluorescent tag circumference ratio in SG were significantly lower than that in OMG, and blueberry did not inhibit their increase in OBG. The active ingredients in blueberries were complex. There may be some ingredients that can affect the osteoid perimeter and the fluorescent tag circumference ratio. More studies were required to explore the active ingredients in blueberries for preventing osteoporosis.

## Conclusion

In conclusion, we have validated the inhibition of rabbiteye blueberry on ovariectomy-induced osteoporosis *in vivo*. The results showed that the rabbiteye blueberries had an effective inhibition in bone resorption, bone loss, and reduction of bone strength of ovariectomized rats, and could improve the BMD, osteogenic activity, and trabecular bone structure. Therefore, we conclude that blueberry might prevent and inhibit ovariectomy-induced osteoporosis, which provides new basis for the clinical treatment of osteoporosis. We showed, for the first time, that rabbiteye blueberries have great potential to accurately, reliably, and safely improve osteoporosis in a rat model of ovariectomy-induced osteoporosis.

The article "Rabbiteye blueberry prevents osteoporosis in ovariectomized rats" was published in 2014. Journal: J Orthop Surg Res.

## Competing interests

The authors declare that they have no competing interests.

## Authors’ contributions

TL participated in the design of this study and performed the statistical analysis. SW carried out the study, together with SO, collected important background information, and drafted the manuscript. ZX conceived this study, participated in the design, and helped draft the manuscript. All authors read and approved the final manuscript.
